# Construction of Digital Economy Trade Security Evaluation System Based on Computational Intelligence

**DOI:** 10.1155/2022/5914561

**Published:** 2022-11-18

**Authors:** Yuqin Zhu, Fengling Wang

**Affiliations:** ^1^School of Economics and Management, Hezhou University, Hezhou 542899, Guangxi, China; ^2^School of Artificial Intelligence, Hezhou University, Hezhou 542899, Guangxi, China; ^3^School of Data Science, City University of Macau, Macao 999078, Macao, China

## Abstract

The upgrading of the digital economy (DE) is crucial to building an intelligent society. The rapid development of computational intelligence in recent years has also brought vitality to the development of the DE. However, with the deepening of international trade, the issue of trade security has become more and more prominent. Therefore, this study aimed to construct a DE trade security evaluation system. For computational intelligence, this study proposes a support vector machine based on improved particle swarm optimization. Such an algorithm can play a key role in the construction of an evaluation system. It is built for the evaluation system. This study selects five indicators of market competitiveness, trade control, trade dependence, market concentration, and trade legal system evaluation. The experimental results of this study prove that the evaluation system proposed in this study is effective. In its test for some countries in the world, the UK trade security index was the highest at 0.582, while China was relatively low at 0.492.

## 1. Introduction

The emergence and progress of new factors of production will often cause great changes in the economic form. From the farming era to the current DE era, the transformation of production factors has undergone three changes. The first change was in the farming era. The key elements of productivity development are land and labor, which are the basic elements of social and economic development. The second revolution was in the age of the big machine factory. The development of science and technology and the emergence of capital have brought great changes to the original key elements of productivity development. At the same time, the substitution of capital for labor has also occurred, and labor has been gradually liberated from complicated work. The third revolution is after entering the twenty-first century, and the economic form has undergone tremendous changes. Data have become another important factor of production besides land, labor, capital, knowledge, etc. The earth has entered the era of interconnection of all things. The economy, society, and information and communication technology (ICT) are intertwined, and nonmaterial production factors such as knowledge, data, and information have entered a stage of explosive growth. In the era of DE, the development of economy and society is manifested as “huge data accumulation.” The development of digital economy has brought about great changes in the mode of production. Countries all over the world have introduced relevant policies to promote the process of digitalization, and the global digital economy is showing a vigorous development trend. Therefore, at present, we should seize the major strategic opportunity period for the development of the global DE, continue to accelerate the pace of digital economic development, and vigorously develop the DE.

At present, the development trend of the DE is unstoppable. At the national strategic level, developing the DE is an important way to promote consumption. It explores the development model of the DE and finds the combination of the DE and the traditional economy. Promoting the development of traditional industries is the proper meaning of developing the DE, but at the same time of development, research on trade security is indispensable.

This study proposes two innovations on the basis of predecessors: (1) for the digital construction of the evaluation system, although the economic research does not use such a complex algorithm, it is very necessary to select an efficient algorithm for the evaluation of DE and the diversification of transaction security indicators. (2) For the construction of the DE trade security evaluation system, this study selects five indicators of market competitiveness, trade control, trade dependence, market concentration, and trade legal system evaluation. These five indicators can well fit the trade security index. This will be mentioned in the subsequent analysis.

## 2. Related Work

Computational intelligence is a branch of machine learning. With the entry into the big data society, there are more and more studies on intelligent learning algorithms, and the research directions are more and more diverse and in-depth. In their study, Olyaie et al. [1] analyzed different artificial intelligence methods, they used different methods to predict the model, and their experimental results showed that the support vector machine model can be used satisfactorily for the estimation of dissolved oxygen [1]. Gomede et al.'s [2] proposed model can develop students' knowledge profiles and can help educators to best position their students in their decisions [2]. Utkarsh et al. [3] show the effectiveness of the method in terms of convergence, adaptability, and optimality relative to centralized and benchmark algorithms through simulations on 30-node and 119-node distributed test systems [3]. Lin et al. [4] demonstrated the feasibility of applying CCA, RBFNs, effective connectivity measures, and D-S theory to help brain-computer interfaces extract informative knowledge from brain signals [4]. Liu and Ting [5] added the application of computational intelligence to music creation and achieved encouraging results. They attempt to provide an overview of computational intelligence techniques used in music creation. First, it is based on the main musical elements considered in the composition, namely, musical form, melody, and accompaniment, and existing methods are reviewed. Second, their research highlights the components of evolutionary algorithms and neural networks designed for music composition [5]. Aldhafferi et al. [6] developed a sensitivity-based linear learning method (SBLLM), which uses ionic radius and dopant concentration as inputs to the model. It trains a two-layer feedforward neural network to estimate the RCP of manganese oxide-based materials [6]. Coyle [7] in turn understands how labor market policies can improve working conditions without limiting the productivity and consumer benefits that digital business models can bring [7].

From the analysis of related research, it can be found that the research and application of computational intelligence mostly stay on the function of the algorithm. Its research on the DE is not very in-depth. In terms of trade security, a lot of blockchain technology is used, and no in-depth research has been done on the evaluation system.

## 3. Computational Intelligence

In 1994, three IEEE international societies related to fuzzy systems, neural networks, and evolutionary computation held the first IEEE World Congress on Computational Intelligence in Orlando, Florida, USA. The topic of discussion was “Computational Intelligence and Imitating Life,” and the concept of “Computational Intelligence” was put forward. It is a new generation of artificial intelligence that emerged after symbolic intelligence, a traditional artificial intelligence. The initial computational intelligence includes three major fields: fuzzy systems, neural networks, and evolutionary computing. In recent years, some emerging methods have also been incorporated into the category of computational intelligence, such as support vector machines, swarm intelligence, rough set theory, artificial immune systems, and DNA computing [8, 9]. Computational intelligence is like a sudden emergence and has been widely used in multidisciplinary fields.

### 3.1. Support Vector Machines

Support vector machine not only has perfect geometric explanation and mathematical form but also has a solid mathematical theoretical foundation based on statistical learning theory (SLT) and the principle of structural risk minimization. It has incomparable superiority in processing small sample data. Support vector machine (SVM) was put forward from 1992 to 1995, and it is the most practical and core part of statistical learning theory.

#### 3.1.1. ERM Principles of Machine Learning

Machine learning is the simulation of human thinking by computer. It first establishes a model through certain rules, then estimates the dependence between the input and output of the solution system according to the existing training samples, and predicts and analyzes the unknown output as accurately as possible, so that the predicted results can reflect the essence of things as much as possible. Machine learning usually consists of three parts. They are the generator *G*, the trainer S, and the learning machine LM, as shown in Figure 1 [10, 11].

The purpose of machine learning is to select the function that can best approximate the response of the trainer from a given set of functions *f* (*x*, *α*) (*x* ∈ *R*^*n*^, *α* is the generalized parameter of the function). This minimizes the expected risk of the trainer. It is assumed that the independent and identically distributed samples are as follows:

(1) $$\begin{array}{c} \left(x_{1},y_{1}\right),\left(x_{2},y_{2}\right),\cdots ,\left(x_{l},y_{l}\right). \end{array}$$

The machine learning problem is to find the optimal function *f*(*x*, *α*_0_) of the above samples in the function set *f* (*x*, *α*). It enables it to minimize the expected risk as shown as follows [12, 13]:

(2) $$\begin{array}{c} R\left(\alpha \right)=\int L\left(y,f\left(x,\alpha \right)\right)\text{d}F\left(x,y\right), \end{array}$$

where *F* (*x*, *y*) is the unknown joint probability distribution function, and *L* (*y*, *f* (*x*, *α*)) is the difference between the learning machine response *f* (*x*, *α*) and the trainer response *y*.

#### 3.1.2. Theory of Generalization

People are most concerned about the generalization ability and learning performance of the learning machine. After studying various types of function sets, statistical theory deduces an important conclusion about the relationship between empirical risk and actual risk, which is called generalization bound, which is an important basis for analyzing the performance of learning machines.

According to statistical learning theory, for all functions in the function set, the following relationship is satisfied with at least 1 − *η* (confidence level) probability between the empirical risk *R*_emp_(*α*) and the actual risk *R* (*α*). It is as follows:

(3) $$\begin{array}{c} R\left(\alpha \right)\leq R_{\text{emp}}\left(\alpha \right)+\frac{B\varepsilon }{2}\left(1+\sqrt{1+4R_{\text{emp}}\left(\alpha \right)/B\varepsilon }\right). \end{array}$$

Formula (3) shows that the actual risk of machine learning consists of the confidence bounds and the empirical risk of the training samples. When the ratio of the VC dimension to the number of training samples is large, even if the actual risk *R*_emp_(*α*) is relatively small, the actual risk *R* (*α*) cannot be guaranteed to obtain a small value. When the VC dimension is relatively large, the system complexity is higher, the *n*/*h* is smaller, and the confidence range is larger. If *R*_emp_(*α*) is used to approximate *R* (*α*), there will be a large error, and the generalization ability of the optimal solution is poor [14, 15]. To obtain a learning system with better generalization performance, it is necessary to achieve a certain balance between the training sample size and the VC dimension. Structural risk minimization is based on this principle.

In Figure 1, *H* is the classification surface, and the two types of samples are represented by hollow points and solid points, respectively. The distance between *H*1 and *H*2 parallel to the classification plane is the classification interval, and *H*1 and *H*2 are determined by the samples closest to the classification plane in the two categories. The corresponding training points on *H*1 and *H*2 are support vectors.

However, this increases the complexity of algorithms (such as neural networks) and increases the VC dimension *h*. The confidence range *φ* (*h*/*l*) then increases, leading to an increase in the actual risk *R* (*α*). This is the overfitting of the learning algorithm, also known as the “overlearning” problem, as shown in Figure 2.

#### 3.1.3. Support Vector Machine Classification Machine

One of the core ideas of SVM [16, 17] is to establish a surface that can correctly separate the two classes and has the largest classification interval, that is, the optimal classification hyperplane (optimal separating hyperplane). It finds the optimal *ω* and *b* and uses the optimal classification hyperplane as the decision surface to maximize the classification margin (margin) between samples. The idea of the optimal classification hyperplane is shown in Figure 3. To maximize the classification hyperplane interval, the optimization problem is constructed, such as follows:

(4) $$\begin{array}{c} \min\frac{1}{2}{\left\|\omega \right\|}^{2}, \end{array}$$

(5) $$\begin{array}{c} \text{s.t. }y_{i}\left[\omega^{T}x_{i}+b\right]-1\geq 0,\;i=1,2,\cdots ,l. \end{array}$$

Minimizing 1/2‖*ω*‖^2^ is to minimize the upper bound of the VC dimension, which realizes the choice of function complexity in the structural risk minimization criterion. When the linearity is inseparable, by introducing a slack variable *ξ* (*ξ* > 0), it is transformed into as follows:

(6) $$\begin{array}{c} \min\frac{1}{2}{\left\|\omega \right\|}^{2}+C\sum_{i=1}^{l}\xi_{1}, \end{array}$$

(7) $$\begin{array}{c} \text{s.t. }y_{i}\left[\omega^{T}x_{i}+b\right]-1\geq 1-\xi_{i},\;i=1,2,\cdots ,l. \end{array}$$

The above optimization problem is transformed into a dual problem by introducing Lagrange multipliers, as shown as follows:

(8) $$\begin{array}{c} \min\frac{1}{2}\sum_{i=1}^{l}\sum_{i=1}^{l}y_{i}y_{j}\left(x_{i}\cdot x_{j}\right)+\sum_{i=1}^{l}\alpha_{1}, \end{array}$$

(9) $$\begin{array}{c} \text{s.t. }\sum_{i=1}^{l}y_{i}\alpha_{i}=0,\;0\leq \alpha_{i}\leq C,i=1,2,\cdots ,l. \end{array}$$

Formula (10) is solved for the pair:

(10) $$\begin{array}{c} \omega =\sum_{i=1}^{l}\alpha_{i}y_{i}x_{i},\;b=y_{i}-\sum_{i=1}^{l}y_{i}\alpha_{i}\left(x_{i}\cdot x_{j}\right). \end{array}$$

Finally, the optimal classification linear discriminant function is obtained, as shown as follows:

(11) $$\begin{array}{c} f\left(x\right)=\mathrm{sgn}\left(\sum_{i=1}^{l}\alpha_{i}\left(x_{i}\cdot x_{j}\right)+b^{*}\right). \end{array}$$

In formula (11), *l* is the number of support vector machines. *α*_*i*_ is the optimal Lagrangian multiplier; *b*^*∗*^ is the threshold.

### 3.2. Improved Particle Swarm Algorithm

#### 3.2.1. Basic Particle Swarm Optimization

In particle swarm optimization (PSO), each solution of the optimization problem corresponds to a particle in the search space. Each particle is an individual consisting of a position vector and a velocity vector [18]. The optimal position (pbest) generated by the particle in motion is shown as follows:

(12) $$\begin{array}{c} p_{i}=\left(p_{i1},p_{i2},\cdots p_{i\;D}\right),\;i=1,2,\cdots ,m, \end{array}$$

where *m* is the number of particles, and *D* is the dimension of the particles.

In each iteration, for each particle, the particle updates itself by tracking two extreme values: one is the optimal solution found by the particle itself, which is called the individual extreme value; the other is the optimal solution found by the whole particle swarm, which is called global extremum. After finding the individual and global extrema, the particle updates its velocity and position according to the following equations:

(13) vik+1=ωvik+cr11pik−xik+cr22pgk−xik,

(14) $$\begin{array}{c} x_{i}\left(k+1\right)=x_{i}\left(k\right)+v_{i}\left(k+1\right), \end{array}$$

where *k* is the number of iterations; *ω* is the inertia weight. To maintain the diversity of the population, *r*_1_, *r*_2_ are random numbers between [0, 1]. *c*_1_, *c*_2_ are the learning factors, also known as the acceleration factors. It enables the particle to have the ability to learn from the excellent individuals in the group and to summarize itself, and at the same time to approach the best point of its own and the best point of the group history.

#### 3.2.2. Improved Particle Swarm Algorithm

This study proposes a new improved particle swarm optimization (IPSO). Its improvement is mainly manifested in two aspects: 1. to facilitate the global search and local search of particles, a strategy of dynamically changing the weight *ω* based on particle distance is proposed. 2. To increase the diversity of particles and avoid the particle swarm from falling into the local optimal solution at the late stage of optimization, chaotic mapping is introduced.

*(1) Dynamic Weight Change Strategy Based on Particle Distance*. This study proposes a strategy for dynamically changing the weight (dynamically changing inertia weight, DCIW) based on the distance between particles and the historical optimal position of the entire population (referred to as particle distance). Under this strategy, the calculation formula of inertia weight is shown as follows:

(15) $$\begin{array}{c} \omega =\omega_{\min}{\left(\frac{\omega_{\max}}{\omega_{\min}}\right)}^{1/\left(1+\varepsilon \cdot k/k_{\max}\right)}. \end{array}$$

In the formula: *ε* is a weight adjustment factor determined by the grain distance. The particle distance of the *i*th particle at the *k*th iteration is defined as follows:

(16) $$\begin{array}{c} d_{i}\left(k\right)=\sqrt{1/D\sum_{j=1}^{D}{\left(x_{ij}\left(k\right)-p_{gj}\left(k\right)\right)}^{2}}. \end{array}$$

Here, *x*_*ij*_(*k*) is the *j*th component of the position vector of the *i*th particle at the kth iteration. *p*_*gj*_(*k*) is the *j*th component of the optimal position vector in the population history at the *k*th iteration. The particle velocity is controlled by choosing the value of *ε* according to the particle distance of each particle, as follows:

(17) $$\begin{array}{c} \varepsilon_{i}\left(k\right)=\varepsilon_{\min}+\left(\varepsilon_{\max}-\varepsilon_{\min}\right)\frac{\left(d_{\max}\left(k\right)-d_{i}\left(k\right)\right)}{\left(d_{\max}\left(k\right)-d_{\min}\left(k\right)\right)}. \end{array}$$

In the formula, *ε*_max_ and *ε*_min_ are the maximum and minimum values of *ε*, respectively, and 15 and 8 are used in this study. *d*_max_ and *d*_min_ are the maximum and minimum grain distances, respectively. When the particle distance *d*_*i*_(*k*) is larger, *ε* will be smaller, and the inertia weight of the particle will be larger. The greater the inertia weight, the greater the particle velocity, which is beneficial to the particle's global search. The smaller the particle distance *d*_*i*_(*k*), the larger *ε* will be, and the smaller the inertia weight of the particle will be. The smaller the inertia weight, the smaller the particle velocity, which is beneficial to the particle's local search. The variation trend of weight *ω* with *ε* is shown in Figure 4.

*(2) It Introduces Chaotic Mapping*. In this study, using the randomness, ergodicity, and regularity of chaotic variables, the chaotic sequence is generated iteratively based on the historical global optimal position gbest currently searched by particle swarm optimization. By adopting the iterative form, the optimal particle position in the chaotic sequence randomly replaces the particle position in the current particle swarm, and many neighborhood points of local optimal solution are generated, thus enhancing the global search ability, getting rid of the attraction of local extreme points, and making the algorithm quickly search for the optimal solution, to improve the search accuracy of the algorithm.

Commonly used chaotic rules are logistic map, Henon map, and tent map. In this study, a two-dimensional discontinuous discrete chaotic dynamic system Lozi formula is selected, such as follows:

(18) $$\begin{array}{c} l_{n}=1-\left(a\left|l_{n-1}\right|+y_{n-1}\right), \end{array}$$

(19) $$\begin{array}{c} y_{n}=b\cdot l_{n-1}. \end{array}$$

In the formula, *n* is the number of iterations; after the parameter *a* > 1.5, it enters the chaotic motion (usually 1.7). The parameter *b* usually takes 0.5, and *l*_*n*_ ∈ [0,1] is the chaotic variable. The research shows that the chaotic method of Lozi map has the advantages of higher solution precision and higher solution efficiency than the commonly used logistic map chaotic method.

### 3.3. Support Vector Machine Based on Improved Particle Swarm Optimization

The appropriate choice of parameters has an important impact on the prediction performance of both classification and regression problems. The parameter optimization problem of SVM is one of the important topics in SVM research.

#### 3.3.1. IPSO-SVM Model Framework

The support vector machine (including classification and regression) training and prediction framework based on IPSO algorithm optimization is shown in Figure 5. The algorithm flow is as follows:

  Step 1: data preparation—all samples are normalized to [−1, 1]. It is divided into two sets of training samples and test samples.
  Step 2: it determines the parameter combination to be optimized according to the support vector machine type to determine the particle swarm dimension.
  Step 3: it determines the particle swarm fitness function according to the support vector machine type.
  Step 4: the training samples are used to train the SVM model with the *k*-fold cross-validation method. The sample set is equally divided into *k* parts, the *k* − 1 part is used for the training process, and the remaining part is used for testing.
  Step 5: it uses the algorithm 3-1 (IPSO algorithm) in Section 3.3 to optimize the parameters of the support vector machine.
  Step 6: it rebuilds and trains the SVM model based on the optimal parameter combination.
  Step 7: it predicts the test sample.

Support vector machine (SVM) is divided into support vector regression (SVR) machine and support vector classification (SVC) machine. The following is a separate study on the integration of the two with IPSO.

## 4. DE and Trade Security

### 4.1. DE

Since the 18th National Congress of the Communist Party of China, China has vigorously promoted the transformation of the mode of economic development. A new round of technological industrial revolution centered on digital, network, and intelligent technology is emerging. As a new economic form, the DE is developing rapidly.

According to the correlation between digital technology and production activities, the DE can be divided into broad and narrow senses. The narrow definition only refers to the information and communication technology industry, including telecommunications, Internet, information technology services, hardware, and software. The broad definition includes both the information and communication technology sector and some traditional sectors combined with digital technology.

Different from the traditional real economy model, the digital economy relies on Internet technology to change the traditional commercial retail model and the development of cross-border e-commerce, effectively improve the efficiency of trade, break the time and space limitation of trade, and have the characteristics of openness and sharing.

By analyzing the important aspects that support the development of digital economy, such as digital infrastructure, digital consumers, digital industry, digital public services, and digital literacy, we can make a comprehensive and accurate judgment on the overall development level of digital economy in an economy.

The CAICT applies the broad definition to digital economic accounting. Its definition structure is shown in Figure 6.

After the 18th National Congress of the Communist Party of China, it has successively launched a series of plans and development strategies such as Network Power and Broadband China to promote the development of the DE. According to the “White Paper on the Development of China's DE (2020),” its details are shown in Figure 7.

With the development of global digital economy entering a new stage of all-round advancement, discussions around international regulations are becoming more and more frequent. The current global economic governance system is dominated by international trade rules and institutional arrangements formed after the Second World War. Western developed countries, led by the United States, have long occupied a monopoly position in formulating and implementing rules, and this order is also reflected in cyberspace. At present, the Internet has become the strategic high point of international competition. Cyberspace breaks the limitation of time and space to form a new living space. The game of rule building on the Internet is becoming increasingly fierce. In other words, in the next stage of the development of the DE, the expansion of cyberspace will mainly be carried out in developing countries and even backward countries. The focus of cyberspace governance will also shift from developed to developing countries. African countries will have the advantage of experience and discourse dominance in cyberspace governance. The governance system of digital economy is still in the exploratory stage, and the change in user structure and number will greatly affect the status and power of the country in cyberspace. The development of digital economy will enable developing countries to reform international rules.

Although domestic and foreign scholars have not formed a unified conceptual identification of the smart industry, however, they all believe that the smart industry has applied emerging information and communication technologies and changed the original production methods. Therefore, it embodies different characteristics from traditional industries. The details are as follows: (1) integration of information technology. The smart industry is based on ICT technology, and in the process of combining with traditional industries, the quality and quantity of traditional industries have been improved; (2) innovation: the application of emerging information technology not only improves production efficiency but also provides more space and possibility for enterprises to innovate in production and accelerates the elimination of industries with low productivity. In addition, the development of smart industry will also promote the emergence of new industries and drive industry innovation; (3) high added value: innovative smart industries will speed up the creation of products. Innovative products must contain greater product value and have higher added value; (4) extensive: smart industries include industries that combine emerging information technology with traditional industries. Therefore, all traditional industries may be combined with emerging information technology. They are all potential smart industries, so they are extensive; (5) ecological: using emerging information technology, smart industry optimizes production methods, reduces environmental pollution, and can greatly reduce ecological damage. It is a sustainable green ecological production method; and (6) wisdom: the final development of the smart industry is to make the industry smart. Its industry situation is shown in Figure 8.

### 4.2. Trade Security

Combining the previous research results and experience, this study argues that, under the current situation of relatively liberalized trade, a country's trade security can be considered to enable a country's trade transactions to proceed smoothly. International trade can play a positive role in promoting the development of a country's economy. At the same time, the impact on international economic fluctuations can also be controlled in an effective state. Then, such a “trade guarantee” can be called trade security.

The competitiveness of an industry is one of the most important factors affecting the development of a country's industry. How the development of an industry is welcomed and has a strong demand in the world fundamentally depends on the competitiveness of an industry's products. Under today's open conditions, international trade links are increasing day by day, and the production and development of any product depend on its competitiveness. For the domestic market of a country, even if domestic products do not go out, foreign products will be imported into the domestic market. So, now domestic competition is also international competition. As the main body of the market, micro-enterprises face the increasingly complex international environment and obtain certain benefits by participating in international competition. It must have and continuously increase the competitiveness of its products, to survive in the fierce international competition market and not be eliminated.

## 5. Construction of the Trade Security Evaluation System

### 5.1. Basic Principles of Construction

It is not easy to establish a scientific and reasonable evaluation index system. For this reason, scholars at home and abroad have put forward a series of principles. On the basis of synthesizing the relevant discussions of domestic and foreign scholars, combined with the characteristics of trade security itself, we propose the following basic principles for constructing the trade security evaluation index system.

### 5.2. Determining Indicator Weights Based on AHP

The Delphi method, also known as expert investigation method, uses back-to-back communications to solicit forecasts from panelists. The judgment of importance contained in the AHP in this study applies the Defer method. The first-level indicators obtained through the scientific expert survey method are shown in Table 1.

### 5.3. Processing of Data

#### 5.3.1. Data Standardization Method

Since there are many index items involved in this study, and the measurement methods are not the same, methods are adopted to standardize various data for the following weighted calculation processing. The min-max standardization used in this study is also called −1 standardization and dispersion standardization.

The conclusion of the trade model that this study is devoted to establishing is the score value of each sub-indicator of trade security. However, the value of some data indicators is not that the larger the value, the higher the score, such as the trade dependence index. The larger the indicator, the more dependent the country's trade is with the exporting country, and if the exporting country experiences economic fluctuations, the country is more likely to be implicated. In this case, this study adopts the standardization index first and subtracts the index from 1 as the final score value. In this way, the processing will be closer to the real level situation.

#### 5.3.2. Standardization of Trade Efficiency Indicators

According to the calculation method of the minimum and maximum values, the *D* C index, the RCA index, and the terms of trade index are standardized separately. According to the expert survey method, these three have the same importance and weight as secondary indicators of trade efficiency. It is then summed up according to the common weight to obtain the data of some of the world's trading countries in Table 2.

#### 5.3.3. Standardization of Trade Control Indicators

The trade structure shows the proportion of a country's service industry to the total GDP, which is a comparison of industries and industries. The content of trade technology products can be considered as a micro-trade structure. Because it represents the proportion of the export of technology products in the total trade volume in an industry, this is an industry-to-industry comparison, which can be understood as a narrow trade structure. The two reflect the changes in trade control from different angles, and the two have the same importance after the expert investigation method. Therefore, after standardizing the indicators of trade structure and trade technology product content, they are summed up with the same weight to obtain Table 3. The data in the table are the trade control index sum of some countries in the world.

#### 5.3.4. Standardization of Trade Dependence Index

The normalization method for trade dependence is similar to the previous two. The difference is that the final trade dependency score of a country needs to be 1 minus this value. Because a country's higher percentage of trade dependence indicates that a country's economy is more dependent on some exporting countries, once an exporting country experiences economic fluctuations or a crisis, the country will receive a relatively strong impact. So, countries with a high trade safety factor should have a smaller percentage. To judge the trade security index more reasonably, this study takes 1 and subtracts the value to obtain Table 4. The data in the table are the trade dependence data of some countries in the world.

#### 5.3.5. Standardization of the Trade Concentration Index

This article uses the trade value of the country's top five largest exporters as a proportion of the country's total trade value. A higher concentration is also not conducive to trade security, so the calculation method is similar to trade dependence. It takes the value of 1 and subtracts this value to get Table 5. The data in the table are the trade concentration index of some countries in the world.

#### 5.3.6. Standardization of Trade Environmental Standards

The importance of the trade environment to trade security has been discussed above. However, it is difficult to use indicators to comprehensively evaluate the trade environment. This study selects the most important and data available indicators that affect the trade environment to evaluate the trade environment. That is the number of cases of trade friction in each country, which will eventually normalize it. Similar to the first two indicators, the higher the number of trade friction cases, the greater the risk to a country's trade security. So, the final result also takes 1 minus the normalized value and finally gets Table 6. The result in the table is the trade environment index of some countries in the world.

### 5.4. Model Data Analysis

Based on the analysis of the above sub-indicators, this section will synthesize the results. On this basis, it does cross-sectional data analysis and time-series data analysis. First, this study assumes that the trade security index *Y* is related to *X*1 (trade efficiency index), *X*2 (trade control index), *X*3 (trade dependence index), *X*4 (trade concentration index), and *X*5 (trade environment index) that have a linear relationship, and the *Y* value is calculated by weighting *X*1 − *X*5.

#### 5.4.1. Cross-Sectional Data Analysis

As can be seen from Figure 9, the trade security index between the UK and the United States leads other countries. They are 0.581 and 0.582, respectively. Compared with China and developed countries, China's trade security situation is relatively weak. The sub-indicators in the UK and the US are average and competitive. Therefore, its trade security evaluation is the two safest countries in the world in 2013.

From the subindices of the UK, its trade concentration index was 0.243. Its trade control index was 0.612, ranking the highest. This shows Britain's strong competitiveness and trade control in foreign trade, especially in service trade and high-tech trade.

Judging from the subindices of the United States, the United States is second only to the United Kingdom in terms of trade competitiveness and trade control, at 0.71 and 0.577, respectively. In addition, the United States' trade dependence index was rated at 0.751. It leads the world and shows its low trade dependence.

India's trade security index was 0.519, leading the indicator among developing countries. Looking at its subindices, India's trade competitiveness index is 0.592. Its trade dependence is relatively low, and both are at a good level. However, its trade control level is 0.323, which is the main factor dragging down its trade security.

Germany's trade security index was at a moderate level of 0.529. Compared with the United Kingdom and the United States, its trade competitiveness advantage is still far away. Germany's trade dependence is also high, of which export dependence is the highest. However, because Germany's exporting countries are relatively scattered, its trade friction is relatively small.

Japan's trade security index was 0.543, and the overall evaluation was good. In terms of subindices, Japan's trade dependence is evaluated as the highest among the selected countries, at 0.777, that is, the lowest trade dependence. Japan's trade competitiveness index was 0.448, which was relatively low, becoming a drag on its trade security.

#### 5.4.2. Time-Series Analysis

Overall, from Figure 10, we can find that China's trade security index decreased year by year from 0.479 in 2000 to the lowest point in 2006 at 0.411. It then continued to rise until 0.491 in 2014. In general, it shows the characteristics of “trade security index U-shaped curve.” The reason for this special phenomenon is that in 2000, China had not yet joined the WTO. China's trade volume is also relatively small, approaching a similar self-sufficiency operating economic model. After joining the WTO in 2001, China's trade volume has undergone tremendous changes. Its growth rate is nearly 55 times. Therefore, when the trade volume was relatively small in 2000, the trade security index was relatively high. Because in an extreme situation where there is no trade volume, trade is absolutely safe. With China's accession to the WTO, the participation in international trade has increased day by day. China has less experience in dealing with various trade frictions and policies internationally. Therefore, when the trade volume increases at the beginning, it will inevitably encounter various international competitions. This makes China's trade security index drop year by year to the lowest point in 2006. However, with the increase and maturity of China's participation in international trade, as well as the maintenance of China's own country's rapid growth, its comparative advantage has gradually emerged. Therefore, the trade security standardization index increased year by year after 2006, until it reached the highest point of 0.491 in 2014. Similar to the Laffer curve of government taxation, the trade security index also exhibits the characteristics of a U-shaped curve with the degree of openness of the country.

## 6. Conclusion

Trade security is related to national economic security. Therefore, the research on trade security cannot be relaxed. Through analysis, we can also find that China's trade security index is temporarily low. However, there is a growing trend, so we still have to pay attention to trade security. This study starts with the analysis of computational intelligence; afterwards, a separate analysis is made of the DE and trade security to obtain corresponding evaluation indicators. Finally, it builds a model for the indicators and proposes a trade security index. Although the results can better show trade security, there are also some shortcomings in this study. In the model construction, there are no classification and discussion on the development of the country. Therefore, future research directions will aim at this.

## Figures and Tables

**Figure 1:** General model of machine learning.

**Figure 2:** Underfitting, fitting, and overfitting.

**Figure 3:** Optimal classification hyperplane.

**Figure 4:** Inertia weight change curve for different *ε* values.

**Figure 5:** Support vector machine based on IPSO parameter optimization.

**Figure 6:** Concept and scope of DE.

**Figure 7:** Scale of China's DE and its proportion in GDP from 2005 to 2018.

**Figure 8:** Schematic diagram of smart industry.

**Figure 9:** Trade security index of some countries in the world.

**Figure 10:** China's 2000–2014 standardized index of trade security.

**Table 1:** List of first-level indicator names.

Index	Name
*X*1	Market competitiveness
*X*2	Trade control power
*X*3	Trade dependence
*X*4	Market concentration
*X*5	Trade legal system evaluation

**Table 2:** Trade efficiency index of some countries in the world.

	Trade benefit index
China	0.415
Germany	0.552
India	0.792
Japan	0.448
Britain	0.808
United States of America	0.710

**Table 3:** Market control index of some countries in the world.

	Market control index
China	0.515
Germany	0.519
India	0.323
Japan	0.535
Britain	0.612
United States of America	0.577

**Table 4:** Trade dependence index of some countries in the world.

	Trade dependence index
China	0.585
Germany	0.528
India	0.695
Japan	0.777
Britain	0.591
United States of America	0.751

**Table 5:** Trade concentration index of some countries in the world.

	Trade concentration index
China	0.536
Germany	0.521
India	0.592
Japan	0.476
Britain	0.218
United States of America	0.293

**Table 6:** Trade environment index of some countries in the world.

	Trade environment index
China	0.39
Germany	0.52
India	0.41
Japan	0.41
Britain	0.53
United States of America	0.42

## Data Availability

No data were used to support this study.
